# Application of Ultrasonic Intelligent Imaging in L-Selectin Regulating Embryo Implantation in Mongolian Sheep Endometrium

This article has been retracted.

**DOI:** 10.1155/2022/3323768

**Published:** 2022-06-16

**Authors:** Changshou Wang, Adong Bao, Qing Hai, Zhengxiang Hu, Xiaoying Bai

**Affiliations:** ^1^Department of Agronomy, Hetao College, Bayannur, Inner Mongolia 015000, China; ^2^Bayannur Forestry and Grassland Bureau, Bayannur Inner Mongolia 015000, China; ^3^Animal Disease Prevention and Control Center, Kezuo Middle Banner, Tongliao, Inner Mongolia 029300, China

## Abstract

In order to explore the practical application of ultrasonic imaging in the pregnancy stage of Mongolian sheep and the role of L-selectin in the embryo implantation process of Mongolian sheep, this paper systematically observed the early embryonic development by B-mode ultrasonic imaging wave diagnostic instrument with 5 MHz rectal probe and detected the expression of sLex and L-selectin in embryonic cells (jar cells) and endometrial cells (RL95-2 cells) by immunoassay to show the role of L-selectin in embryonic adhesion. The results were as follows: the correct rate of fetal sex determination by ultrasound imaging increased with the increase of pregnancy days and reached 93% at 84 days; sLex/L-selectin on the surface of Jar/RL95-2 cells is involved in the adhesion between embryo and endometrium; and when the concentration of L-selectin was 30 *μ*g/ml, the implantation success rate of fertilized eggs and embryos was the highest, reaching 95%. It is proved that ultrasonic intelligent imaging exploration can summarize the imaging characteristics of the early development law of sheep fetus, which provides a basis for B-ultrasound to monitor fetal growth and predict fetal age. While discussing the molecular mechanism of implantation, it provides a new idea and means for the clinical intervention of contraception and pregnancy assistance with oligosaccharide as the target.

## 1. Introduction

Livestock embryo transfer technology has developed from the experimental stage after the 1980s to 1990s to the application of livestock production, which has become a major revolution in livestock breeding and improvement technology. Sheep embryo transfer technology refers to the use of improved breeds or excellent individual ewes as donors for superovulation, so that they can produce more embryos and take the varieties or individual ewes with poor production performance as recipients. The embryos produced by the donor are transferred into the recipient's uterus by surgical method, and the fetus of excellent individuals is conceived by the belly of poor ewes, so as to achieve the purpose of rapidly expanding the offspring of good breeding sheep. The reproduction speed of purebred sheep can be greatly accelerated by carrying out sheep embryo transfer technology [1]. Due to the current shortage of purebred sheep in China, the market price of each purebred sheep is tens of thousands of Yuan. Embryo transfer technology can improve the reproduction efficiency of purebred sheep several times or more than ten times. As an effective way to speed up the reproduction speed of improved sheep, embryo transfer technology can obtain good economic and social benefits, and its application prospect is very broad. Among the factors affecting the production efficiency of raising sheep, variety is the primary factor. The application of excellent sheep breeds is the basis for improving the production level of sheep and promoting the development of sheep industry [2]. The growth performance and meat production performance of some excellent foreign sheep breeds are better than those of domestic local breeds. However, due to the expensive introduction of breeding sheep, low reproductive rate and, long reproductive cycle, they cannot be popularized rapidly. Young sheep aged 2-5 years old with good phenotype, high production level, stable heredity, healthy physique, normal estrous cycle, no reproductive tract diseases, and normal reproductive history of 1-2 fetuses were selected as donors [3]. The donor and recipient sheep must be selected and kept in place 3~4 months before the operation, and the epidemic disease vaccination, necessary epidemic disease monitoring, and insect repellent shall be done well, and the feeding shall be strengthened from 2 months before the operation. Especially in the treatment of donor sheep, if the feeding management is not in place, it will cause nonovulation or corpus luteum to form white body and affect embryo quality and nonfertilization of embryos [4]. It is suggested to eliminate the donor sheep that are too thin and avoid the waste of hormones and human and material resources. The sheep also suffer from poor embryo production effect and slow surgical recovery. Select an excellent donor and acceptor. Empty ewes with large size, no reproductive tract diseases, high milk yield, and strong lactation ability are selected as the acceptor. The acceptor sheep are 2~5 years old and have a history of normal reproduction of 1~2 fetuses. It is suggested to eliminate too thin recipients. The embryo transfer rate of too thin recipients is low, resulting in the waste of hormones, manpower, and material resources. In addition, before and after embryo transfer, how to promote the success rate of transfer and judge whether embryo implantation has become a key issue [5].

## 2. Literature Review

Sui et al. believed that after embryo transfer, pregnancy diagnosis should be made as soon as possible to determine the sheep without pregnancy, and timely measures should be taken to make them pregnant, which is of great significance for protecting the fetus, reducing empty pregnancy, shortening the litter interval of ewes, and improving the reproductive rate of sheep [6]. Pillarisetti et al. believe that in practice, the most commonly used pregnancy identification method is to test the estrus of rams to observe whether the transplanted sheep return to estrus. If they do not return to estrus, they are pregnant, and if they return to estrus, they are not pregnant. Generally, they test estrus continuously for 2-3 estrus cycles. This method has a good effect on ewes with normal estrus, and the accuracy is more than 90%. It is not applicable to false pregnant sheep without pregnancy and estrus and those who have estrus after pregnancy, but this phenomenon occurs less in sheep production [7]. Labuda et al. believe that after pregnancy, ewes have vigorous metabolism, increased appetite, and improved digestive function, which are manifested in weight gain, glossy coat, docile temperament, cautious and stable action, etc. these phenomena can be used as important indicators for external observation. In actual production, the number of no return cases is often higher than the actual number of conceived babies. To solve this problem, the following methods can be adopted for further inspection [8]. Zhang et al. believed that ultrasonic detection method is to use the reflection of ultrasonic wave for pregnancy examination. This method is generally used at 6 weeks of estrus, and the accuracy rate is about 98%. Ultrasonic diagnosis is a physical examination method that closely combines the physical characteristics of ultrasound with the acoustic characteristics of animal tissue structure. The specific method is to keep the ewe standing in the seminiferous frame, fix the neck with a rope, and examine it in two ways: rectum and in vitro. First from the rectum, when the rectum cannot be accurately examined, use in vitro examination. During rectal examination, first take out the resident feces in the rectum, apply the coupling agent on the probe, bring it into the rectum by fingers, send it to the front and back of the pelvic entrance, and scan it at 45°-90° downward. In in vitro examination, it is mainly in the hairless area on the inner side of the roots of the two strands or on both sides of the breast without shearing. After the probe is coated with coupling agent, it is scanned by sticking the skin to the direction of the uterus at the entrance of the pelvic cavity, and typical images are selected for photography and video recording [9]. Mohammadkhani et al. believed that the content of progesterone in the blood of ewes increased significantly after pregnancy. According to this characteristic, the ewes were diagnosed for early pregnancy, that is, measured by fluorescence spectrophotometry 20 days after transplantation. The progesterone content per milliliter of plasma in sheep was more than 1.5 *μ*g, the accuracy of infertility was 100%, and the accuracy of pregnancy was 93%. The progesterone content per milliliter of milk of dairy goats is greater than or equal to 8.3 *μ*g, the accuracy of infertility is 100%, and the accuracy of pregnancy is 90%. The accuracy of infertility and pregnancy was 100% and 98.6% in sheep when the content of progesterone in plasma per milliliter was greater than or equal to 3 *μ*g. The plasma progesterone content of goats per milliliter is greater than 3 *μ*g, and the pregnancy accuracy is 86% [10]. Luo et al. believe that after ewe pregnancy, the embryo, placenta, and maternal tissue produce prolactin or enzyme chemicals, respectively, and their content increases significantly in a certain period after pregnancy. Some substances have strong antigenicity and can stimulate the immune response of ewe body. Pregnancy can be identified through some physical and chemical properties of antigen antibody binding reaction, such as agglutination reaction and precipitation reaction. Generally, the specially prepared anti pregnancy serum can be used to check whether the ewes 10-15 days after mating are pregnant [11]. After Fan et al. first used the ultrasound imaging technology to diagnose sheep pregnancy, many scholars used it to predict gestational age and gestational period [12]. For example, Zhong and others used it to measure placental diameter to predict gestational age. They believed that there was a positive correlation between gestational age and placental growth, but they found that the placental diameter had developed to the maximum by 80 d of pregnancy [13]. Tenorio-Chávez and others used it to measure the biparietal diameter (BPD) of the fetal skull to predict fetal age [14] In addition, Reichert and others also used it to monitor the effects of forage poisoning on sheep fetal development, such as abortion and teratogenesis. Although the above prediction has gone deep into the study of fetus itself, there is no report on the observation of sheep fetal development system [15].

Based on this, this experiment is to observe the early development law of sheep fetus through systematic tracking and exploration on the basis of ultrasonic imaging in the diagnosis of early pregnancy of sheep, in order to provide useful data for the feeding and management of sheep during pregnancy, the monitoring of embryo growth, and development and the diagnosis of related diseases (Figure 1).

## 3. Research Methods

### 3.1. Ultrasonic Imaging Exploration

The Alokassd210dx-ii ultrasonic diagnostic device (referred to as B-ultrasound, with rectal probe), frequency 5 MHz, with photographic and video equipment, was used

9 Mongolian and hybrid pregnant ewes of 1~2 generations, 4 at 15~18 days after mating, and 5 at 30~38 days of pregnancy were included. Ewes stand or lie on their sides, exclude feces stored in the rectum, take the probe into the rectum by fingers after applying coupling agent, and scan it to the front of the bladder, down and at 45 on both sides, observe the fetal body, fetal heart, fetal viscera, fetal movement, placenta, etc., and select typical images for photography and video recording [15].

### 3.2. Effect of L-Selectin on Embryonic Cells

#### 3.2.1. Cell Culture

RL95-2 cells were cultured in the DMEM/F12 (1 : 1) medium (containing 10% fetal bovine serum, 5 g/ml insulin, 100 IU/ml penicillin, and 100 g/ml streptomycin), and jar cells were cultured in the RPMI1640 medium. Culture conditions are as follows: 37°C, volume fraction 5% CO_2_, and 90% saturated humidity.

#### 3.2.2. Cell Transfection

The cells were spread on 6-well plates and transfected with liposome 2000 when they grew to 70%-80% fusion. Take 4.0 *μ*g FUT7 overexpression vector and gently mix it with 250 *μ*l medium (no serum, no double antibody); 10 *μ*l liposomes were gently mixed with 250 *μ*l DMEM/F12 medium (serum-free, double antibody free) and incubated at room temperature for 5 min. Mix the above two liquids evenly and incubate them at room temperature (25°C) for 20 minutes to form DNA and liposome complex. Add the cell pores to be transfected, culture for 4 hours under the conditions of 37C, volume fraction of 5% CO_2_ and 90% humidity, and add 1 ml of DMEM (containing volume fraction of 20% fetal bovine serum) to each well. After transfection, the cells were cultured for 48 hours under the same conditions [16].

#### 3.2.3. Cell Adhesion Test

Endometrial cells (RL95-2) are laid in the culture hole with cover glass in advance, and the cells climb and grow. After the cells grew to 90% fusion, jar cells were collected, counted, and added to RL95-2 cells for coculture for 1 h. Take out the cover glass containing RL95-2 and jar cells, invert it into a centrifuge tube containing PBS, and centrifuge at 1000 r/m for 5 min. Take out the cover glass and collect and count the nonadherent jar cells. Calculate the adhesion rate of embryonic cells. The adhesion rate = (number of jar cells adhered/number of jar cells added) × 100%.

### 3.3. Role of L-Selectin in Embryo Transfer

Different concentrations of L-selectin were incubated with Mongolian sheep fertilized eggs and then transferred to the uterus of healthy age recipient ewes, and then the embryo implantation was detected by ultrasonic imaging to analyze the effect of L-selectin on Mongolian sheep embryo implantation [17].

## 4. Result Analysis

### 4.1. Results of Ultrasonic Imaging Detection of Pregnant Ewes

The fetal body reflex is an oval light mass with weak reflection in the dark area of the uterine horn. The body length is about 0.6 cm at the first 19 days after mating and increases to 1 cm at 21 days. The measurement was carried out until the 43rd day of pregnancy, and then the measurement was stopped because the full length of the fetus could not be displayed. The fetal body increases with the increase of pregnancy days. It takes about 7 days for the fetal body to grow by about 1 cm from 28 to 41 days. It seems to grow faster after 40 days of pregnancy.

Fetal heart beat can be observed on the 20th day of pregnancy. After 43 days of pregnancy, due to fetal growth, fetal heart beat can be seen only when fetal chest is scanned. Fetal chest depth was 2.7 cm at 58 d and 4.6 cm at 83 d. Fetal heart area is 1.8 cm × 1.5 cm at 68 d 2 cm, 2.1 cm × 1.2 cm on 76 d, and 2.5 cm wide on 83 d [18].

According to whether there is scrotal reflex, due to fetal movement, fetal position is difficult to fix, and it is difficult to judge the gender. Three cases were randomly judged in the test, one case on the 47th and 61th days of pregnancy. A convex weak reflex was observed between the roots of two hind limbs, which was considered the scrotum. It was judged as a male lamb, and the postmortem examination was in accordance with [19]. One case was judged as a male lamb according to the convex reflection at 52 d, and the sheep scanned the part at 89 d, but no convex weak reflection was found, so it was judged as a female lamb, and it was confirmed as a female lamb after autopsy. The specific results are shown in Figure 2. The correct rate of fetal sex determination by ultrasound imaging increased with the increase of pregnancy days and reached 93% at 84 days.

The placenta was first detected on the 30th day of pregnancy. There was a small flat oval bulge on the uterine wall, about 0.3 cm long. From the first detection of the placenta on the 30th day of pregnancy to the 77th day of pregnancy, it increases with the increase of the number of days of pregnancy, as shown in Figure 3. The size of placenta detected after 77 d did not increase with the increase of gestational days. The umbilical cord reflex and umbilical artery pulsation were found at 33 d of pregnancy. The umbilical cord diameter increased with the increase of pregnancy days. On 89 d, four lumen umbilicuses were detected, that is, the cross-section of umbilical cord showing the lumen of four vessels of umbilical cord at the same time, which is 1.5 cm × 1.3 cm. The fetal urachal tube and bladder connected to it were observed [20].

### 4.2. The Role of L-Selectin in the Adhesion between the Embryo and Endometrium

Under normal conditions, the adhesion rate between jar cells and RL95-2 cells is 69.7 ± 2.6%. When jar cells are blocked with sLex antibodies of 0.05 *μ*g/ml, 0.5 *μ*g/ml, and 5 *μ*g/ml, respectively, the adhesion rates between JAR cells and RL95-2 cells are 64.9 ± 1.1%, 53.8 ± 4.4%, and 35.3 ± 1.5%, respectively, that is, after sLex antibody treatment, the adhesion rate between jar cells and RL95-2 cells decreases in a dose-dependent manner [21]. When the antibody concentration was 30 *μ*g/ml, the adhesion rate was 40.3 ± 3.68% (*P* < 0.01), as shown in Figures 4 and 5.

After blocking RL95-2 cells with the sLex antibody, the adhesion rate between jar cells and RL95-2 cells decreased. When the concentration of sLex antibody was 5 *μ*g/ml, the inhibition degree was the most obvious (35.3 ± 1.5%). The difference was statistically significant (*P* < 0.01) [22]. RL95-2 was blocked with the L-selectin antibody. When the concentration of L-selectin antibody was 30 *μ*g/ml, the adhesion rate was 42.6 ± 2.4% (*P* < 0.01). Compared with the untreated group (68.9 ± 1.4%), the adhesion rate decreased significantly, as shown in Figures 6 and 7.

In order to further explore the role of sLex/selectin adhesion system in embryo implantation, the role of sLex in embryo implantation was studied by regulating the synthesis level of sLex [23]. Both in vivo and in vitro studies show that FUT7 is the key enzyme for sLex synthesis. After transfection of FUT7 overexpression vector into jar cells or RL95-2 cells, the expression of FUT7 increased, and the synthesis of sLex oligosaccharide antigen on the cell surface increased. Cell adhesion experiment showed that after jar or RL95-2 cells were transfected with FUT7 overexpression vector, compared with the nontransfected group (68.9 ± 1.4%), the adhesion rate between jar and RL95-2 cells increased (86.6 ± 3.0%, 84.3 ± 1.9%). After two kinds of cells were transfected with the FUT7 overexpression vector at the same time, the adhesion rate between jar and RL95-2 cells increased most significantly (89.4 ± 1.2%) (*P* < 0.01), as shown in Figure 8.

In conclusion, sLex/L-selectin on the surface of JAR/RL95-2 cells is involved in the adhesion between embryo and endometrium.

### 4.3. Effect of L-Selectin on Embryo Implantation

After incubation with Mongolian sheep fertilized eggs with different concentrations of L-selectin, they were, respectively, transplanted into the uterus of healthy age recipient ewes, and then the implantation of embryos was detected by ultrasonic imaging. The results are shown in Figure 9.

When the concentration of L-selectin is 30 *μ*g/ml, the implantation success rate of fertilized eggs and embryos is the highest, reaching 95% [24].

## 5. Conclusion

The results of this experiment have a preliminary understanding of some regularity of the early development of sheep fetus. Although there are few data and need to be further studied in the future, it has been explained that ultrasound imaging is a good method to visually study the fetus and its physiological activities. This paper preliminarily summarizes the imaging characteristics of the early development law of sheep fetus, which provides a basis for monitoring fetal growth by B-ultrasound and predicting fetal age. For the prediction of gestational age and gestational period, it is more scientific to make a comprehensive judgment when measuring the fetal body length, head length, and placental size, combined with the characteristic changes of fetal development in different stages of pregnancy. During the implantation window, embryonic jar cells express sLex oligosaccharide antigen, and endometrial RL95-2 cells express L-selectin. The mutual recognition of sLex and L-selectin mediates the adhesion between mother and fetus. At the same time, jar cells express L-selectin, and RL95-2 cells express sLex. The combination of the two also plays a biological function in the process of embryo implantation, that is, sLex/L-selectin adhesion system plays a role in the two-way recognition of sLex and L-selectin between the mother and fetus. While exploring the molecular mechanism of implantation, this study provides a new idea and means for the clinical intervention of contraception and pregnancy assistance targeting oligosaccharides.

## Figures and Tables

**Figure 1:** Ultrasonic imaging method.

**Figure 2:** Success rate of ultrasound imaging in detecting gender.

**Figure 3:** Changes in placental growth.

**Figure 4:** Effect of L-selectin on adhesion of jar cells to RL95-2 cells (sLex Ab).

**Figure 5:** Effect of L-selectin on adhesion of JAR cells to RL95-2 cells (L-selectin Ab).

**Figure 6:** Effect of L-selectin on the adhesion of RL95-2 cells to jar cells (sLex Ab).

**Figure 7:** Effect of L-selectin on the adhesion of RL95-2 cells to JAR cells (L-selectin Ab).

**Figure 8:** Effect of FUT7 on the adhesion rate between jar and RL95-2 cells.

**Figure 9:** Effect of L-selectin on embryo implantation.

## Data Availability

The data used to support the findings of this study are available from the corresponding author upon request.
